RETRACTED

# TNF-like weak inducer of apoptosis / nuclear factor κB axis feedback loop promotes spinal cord injury by inducing astrocyte activation

**DOI:** 10.1080/21655979.2022.2068737

**Published:** 2022-05-03

**Authors:** Dexiang Ban, Peng Yu, Zhenyang Xiang, Yang Liu

**Affiliations:** Department of Orthopaedics, Tianjin Medical University General Hospital, Tianjin, China

**Keywords:** Spinal cord injury (SCI), TWEAK, NF-κB, astrocytes, autophagy

## Abstract

Non-canonical signaling pathways have been proved to act as potent sites of astrocytes osmotic expanding or proliferation, which promotes the regeneration of axons in areas with non-neural spinal cord injury (SCI). However, the relevant signal pathway that induces autophagic cell death in astrocytes and its function relative to the TNF-like weak inducer of apoptosis/nuclear factor κB (TWEAK/NF-κB) axis remains elusive. The SCI model was established by vertically striking the spinal cord according to Allen’s model. Astrocytes and neuronal cells were prepared from spinal cells extracted from spinal cord tissues of SCI or normal C57BL/6 newborn mice. After co-culturing astrocytes and neurons, cell viability and autophagy were determined by CCK-8, transmission electron microscopy (TEM), and western blot. The expression of TWEAK, NF-κB and inflammatory cytokines was confirmed by qRT-PCR, western blot, Immunofluorescence and ELISA assay. Chromatin immunoprecipitation (CHIP) was used to evaluate the interaction between TWEAK and NF-κB. Our results demonstrated that knockdown of TWEAK and NF-κB inhibited secretion of high levels of TNF-α/IL-1β, partially counteracted by adding Rap. TWEAK/NF-κB was the positive correlation feedback loop regulating the proliferation and autophagy of astrocytes involved in SCI. Moreover, restraining the excess growth of astrocytes was beneficial to the growth of neurons. Collectively, our findings illustrated that the TWEAK/NF-κB pathway might act as a positive modulator of SCI by inducing astrocyte activation, shedding new insights for SCI treatment.

## Introduction

Spinal cord injury (SCI) is a severe central nervous system disorder that usually results in permanent impairment of the function of the injured sub-segmental nerves [1,2]. Increasing attention has been paid to the functions of glial cells in the central nervous system. The astrocyte, a crucial glial cell in the central nervous system, is involved in various neurophysiological and pathological processes of the central nervous system. When SCI occurs, the injured local astrocytes are activated, resulting in reactive cell proliferation and hypertrophy. Eventually, dense glial scar forms, thus affecting the regeneration and repair of SCI [3]. Previous studies have suggested that astrocytes may hinder neurological recovery and promote the progression of SCI after central nervous system injury [4].

RETRACTED

Astrocytes play a significant role in the regular spinal cord, accounting for about 90% of the cells in the central nervous system, and play an essential role in the regular spinal cord in two main ways. For one thing, astrocytes provide structural support and nutrition for neurons; in the central nervous system, most space between neurons and their processes is filled with astrocytes which play a structural supporting role for neurons. For another, astrocytes synthesize and secrete a variety of neuroactive factors at low levels under certain physiological conditions, such as TNF-α, IL-1β, INF-γ, TWEAK and other significant factors of neural inhibition [5–7]. These cytokines work together to nourish and maintain the survival of neurons, promoting the growth of neurites to a certain extent. Satake *et al*. have confirmed that these neurotrophic factors are secreted in normal spinal cord tissues and secreted by early astrocytes in SCI, thus promoting the regeneration and repair of axons [8]. In addition, these factors are also involved in the division and differentiation of nerve cells, blood cell generation, immune regulation, and inflammatory response.

Autophagy is a conserved catabolic process whereby damaged organelles and proteins are sequestered in double membrane vesicles called autophagosomes [9]. Under physiological and pathological conditions, autophagy can be activated as a protective mechanism to maintain or restore intracellular homeostasis [10]. Conversely, once the balance is lost, autophagy can also lead to cellular damage such as mitochondrial and lysosomal dysfunction, endoplasmic reticulum damage, and even programmed cell death [11]. Enhanced autophagy after SCI may weaken the expression of downstream molecules involved in neuronal apoptosis, including cleaved Caspase-3 and Bax, leading to dissociation of the Bcl-2/Beclin-1 complex. Therefore, determining the neuroprotective mechanisms involved in autophagy mediated neuronal survival, particularly the interplay between glial activation and autophagy, may provide new therapeutic strategies for SCI [12].

The TNF receptor family modulates numerous critical biological processes related to tissue homeostasis and diseases, including cellular apoptosis, differentiation, and inflammation [13]. Spinal astrocytes secreted TNF-α, which damaged neurons and promoted eukaryotic NF-κB activating, causing cells to produce oxygen-free radicals such as nitric oxide (NO). NO affected the excitability of nerve cells, promoting sensory conduction, thus promoting inflammation and pain [14,15]. NF-κB was a transcription factor regulating the expression of massive genes involved in inflammation responses, autoimmune response and cell proliferation [16]. In addition, misregulation of the NF-κB signal transduction pathway was observed in various human cancers, especially those of lymphoid cell origin [17].

RETRACTED

TWEAK, a member of the TNF superfamily, is expressed by glial cells inducing astrocyte proliferation and production of cytokines and has also been identified as an essential mediator of inflammation. Previous reports have revealed that TWEAK had a pro-inflammatory effect on human astrocytes in culture, indicating its potential role in central nervous system inflammation. Under normal conditions, relative low-level expression of TWEAK has been demonstrated in previous reports. However, relative expression of TWEAK was up-regulated under pathological conditions including in a neonatal hypoxic mouse model [18,19]. Moreover, recent studies had demonstrated that TWEAK and Fn14 were over-expressed in gliomas with a high level of NF-κB activation, suggesting that the TWEAK-NF-κB axis might serve as a potential target of neuroregulatory mechanisms in a context-specific manner [20].

In this study, we aimed to explore the effect of the TWEAK-NF-κB axis on SCI and investigated the role of the pro-inflammatory TWEAK/NF-κB pathway in astrocytes in a mouse model of SCI. We assumed that the TWEAK/NF-κB pathway promotes spinal cord injury by inducing astrocyte activation. The findings of this study may provide a new idea for the treatment of spinal cord injury.

## Materials and methods

### Animals and ethics statement

A SCI mouse model was established for the regulation mechanism analysis as previously reported [21]. Eight-week-old C57BL/6 mice were used (Model Animal Research Center of HIBIO Co., Ltd, Hangzhou, China). They were fed under pathogen-free conditions at room temperature and a standard laboratory diet with free access to regular water. In addition, all experimental groups were sex-matched on average for all histological analyses to avoid sex-dependent influences. All procedures were approved by the Animal Ethic Committee of Hangzhou HIBIO Co., Ltd.

To explore the effect of TWEAK-NF-κB axis during SCI, histopathology was conducted by Hematoxylin and Eosin (HE) staining and Masson staining. The mice were randomly divided into the following groups: Control, SCI, SCI+Lv-sh-NC (negative control), SCI+Lv-sh-TWEAK, SCI+Lv-sh-NC, SCI+Lv-sh-NF-κB. The lentivirus vectors expressing sh-NC, sh-TWEAK and sh-NF-κB (10^5^ plaque-forming units) were provided by GenePharma (Shanghai, China) and were injected into the intrathecal space of mice using a glass micropipette.

RETRACTED

### Hematoxylin and eosin (HE) and Masson staining

The histological analysis of mouse spinal cord injury was performed using HE and Masson staining. Briefly, mouse spinal cord tissues were embedded in paraffin, horizontally cut into 8 μm slices. Then HE staining and Masson Trichrome staining (Boster, Wuhan, China) were performed after deparaffinization with xylene and hydration according to the manufacturer’s protocol. The images were taken under a light microscope [22].

### Astrocyte culture

The spinal cord tissues were collected at 3 days post-SCI. Spinal cord tissues were removed by opening the spinal canal and digested repeatedly with 0.125% trypsin. Then the spinal cells were collected by centrifugation. Primary spinal cells were harvested from mice spinal cord underwent gentle agitation in 0.25% trypsin-Ethylene Diamine Tetraacetic Acid (EDTA) for 20 minutes. Mice spinal cord tissues were triturated gently to prepare the single-cell suspension, which was filtered through a 70-µm nylon mesh cell strainer to wipe off debris. Astrocytes were prepared from spinal cells in suspension and maintained in 5 ml of DMEM/F12 with 50 U/ml penicillin and 50 µg/ml streptomycin, 10 mM HEPES, and 10% fetal calf serum (FCS). Astrocyte cells were separated from confluent mixed glial cultures to 97% purity using magnetic bead technology. The cells were seeded into poly-L-lysine (Sigma, Saint Quentin Fallavier, France) (12 Ag/ml)-coated flasks at the density of 2 × 10^5^ cells/cm^2^. After growing overnight in the growth medium in a 37°C incubator, astrocytes were split by the magnetic bead technology for different experimental treatment conditions in the following day [18].

### Neuronal cell culture

Normal C57BL/6 newborn mice were killed and immersed in 75% ethanol for disinfection. Similarly, the spinal canal was opened, and the spinal cord tissue was removed. After the spinal cord was cleaned and cut into small pieces, they were digested for 30 minutes by 0.125% trypsin repeatedly. The tissue blocks were fully settled to the bottom of the tube after washing 3 times. Finally, 1 ml of inoculation solution was used for suspension. The tissue blocks in the suspension were repeatedly blown (Pasteurized straw) with a moderate force. Next, the cells were collected by centrifugation. About 5 ml of supernatant containing single-cell suspension was collected in a culture flask to re-suspend the cells in the inoculation solution. Finally, 1 × 10^7^ cells were inoculated in a 6-well culture plate for 24 hours until the cells adhered to the wall. To observe the growth status of neurons, cells should be cultured in a full culture medium for at least 3 days [18].

RETRACTED

### Short hairpin RNA (shRNA): design, construct, and validation of gene interference

Herein, we introduced shRNA into spinal cord cells through infection with viral vectors, which allows for a stable construct of shRNA and interference of the targeted gene; We selected the shRNA target sites and designed shTWEAK/NF-κB sequencing through shRNA hairpins, and verified the cellular mechanism of RNA interference. After the shRNA plasmid was prepared and introduced into the cells, it effectively confirmed interference by quantitative Real-Time PCR analysis (Bio-Rad, USA). PCR was performed with the mTWEAK and NF-κB oligonucleotides: 5′GATCCGCAGGGAAGACCC3′ and 5ʹCAGAAACTCATCTCTGAAGA3′, respectively [23].

### Short hairpin RNA transfection

According to the manufacturer’s protocol, the isolated primary spinal cells were used for the shRNA transfection with EntransterTM-R4000 (Engreen Biosystem, Beijing). Spinal cord cells were plated at 2 × 10^5^ cells/well in 6-well plates one day before transfection. Firstly, 3.3 μg shRNA and a certain amount of opti-mem serum-free diluent were thoroughly mixed to form an RNA diluent with a final volume of 25 μL. Next, a total of 1.5 μL entranster-R4000 and 24 μL serum-free dilution were added to make a dilution of entranster-R4000 with the final volume of 25 μL. Finally, the transfection complex was prepared by mixing the entranster-R4000 diluent and RNA diluent. The complex diluent was aspirated with a sampler more than 10 times thoroughly and stood at room temperature for 15 minutes. Next, the 50 μL transfection complex was dripped onto 0.45 ml full-medium, which contained 10% serum and antibiotics. Then the culture dish was moved back and forth repeatedly. At last, cells were transfected with shTWEAK and shNF-κB for 48 hours [19].

### Co-culture model of astrocytes and neurons

To explore the effect of TWEAK/NF-κB gene knockdown on co-cultured neurons, co-cultures of neurons and astrocytes were grown in the transwell system with a 0.4 μm pore size. Neuronal cells were seeded in the upper compartment of the 6-well transwell system, in which 5 × 10^5^ astrocytes were inserted cultured in the lower compartment. Cells were cultured in DMEM with 10% fetal bovine serum, 50 IU/mL penicillin and 50 pg/mL streptomycin, 2 mM L-glutamine and 1% sodium pyruvate. In this methods, the neurons and astrocytes were physically separated while the medium was intermixed [24].

### Quantitative reverse transcriptase polymerase chain reaction (qRT-PCR)

Total RNA was extracted using TRIzol reagent (EX1880-100 ml; G-Clone, Beijing, China), followed by measuring the concentrations of RNA using a spectrophotometer. Then, RNA was reverse transcribed into cDNA using Hifair® III 1st Strand cDNA Synthesis SuperMix Kit (11141ES10; YEASEN, Shanghai, China) as per the instructions. Afterward, PCR amplification reaction was performed using Hifair® III One-Step RT-qPCR SYBR Green Kit (11143ES50; YEASEN, Shanghai, China) on ABI 7500 PCR system (Applied Biosystems, USA). The PCR thermal cycles were as listed: initial denaturation at 95°C for 10 minutes, 35 cycles of 95°C for 10 seconds and 65°C for 15 seconds. β-actin functioned as the internal control, and the related gene expression was measured by the 2^−ΔΔCT^ method [25]. The primers information was listed in Table 1.

RETRACTED

**Table 1.** The sequences of all primers used in qRT-PCR

Gene name	Primer sequence
NF-κB	Forward: ATGGCTACTATGAGGCTGACCTC
	Reverse: TGCCGATGCACATCAGCTTGAG
TWEAK	Forward: GGAACACTCCAAAAACAGACCT
	Reverse: CCACCACTGGGTATTGAGTAGAA
β-actin	Forward: GTCCCTCACCCTCCCAAAAG
	Reverse: GCTGCCTCAACACCTCAACCC

### Transmission electron microscopy (TEM) analysis

Cells were digested with 0.25% trypsin and made into cell suspension. The cell suspension was centrifugated at 4°C, 2000 rmp for 5 min. Then the pre-cooled 2.5% glutaraldehyde was slowly added dropwise along the tube wall and fixed overnight at 4°C. The samples were dehydrated in a gradient of 50%->70%->80%->90%->95%->100%->100% ethanol for 10–20 min for each step. Finally, Under transmission electron microscopy, images were collected to observe the ultrastructure of the samples [26].

### Cell viability assay

Astrocyte viability assays were performed with Cell Counting Kit-8 (CCK-8) (Mibio, Shanghai, China). Firstly, 100 μL of target astrocyte suspension with the density of 2 × 10^5^ cells was prepared in a 96-well plate and pre-cultured in the incubator at 37°C for 24 hours. Next, 10 μL of CCK8 solution was then added to each well carefully to avoid forming bubbles affecting the optical density (OD). Finally, the absorbance was detected with the microplate reader (Molecular Devices, America) by spectrophotometry at 450 nm.

### Nuclear and cytoplasmic protein extraction

We extracted nuclear protein and cytoplasmic protein from cultured cells using a Nuclear and Cytoplasmic Protein Extraction Kit (Beyotime, Shanghai, China). Cells were washed twice with PBS, and the protein extraction reagent A was then added. The mixture was vortexed for 5 seconds and incubated on ice for 15 minutes. Next, 10 μL of extraction reagent B was added, vortexed and put on ice for two minutes. Then we vortexed the mixture for 5 seconds with maximum speed and centrifuged it at 4°C for 5 minutes. The supernatant was immediately absorbed into a precooled plastic tube to obtain the extracted cytoplasmic protein. Similarly, the extracted nuclear protein was obtained by immediately absorbing the supernatant into a pre-cooled plastic tube according to the kit operation instruction [27].

RETRACTED

### Western blot assay

Astrocyte cell lysates were prepared using modified RIPA buffer and normalized for equal protein loading amounts using a Bradford protein assay. The extracted protein was loaded on the polyacrylamide gel and then transferred onto a polyvinylidene fluoride (PVDF) membrane. The PVDF membrane was blocked with 5% nonfat milk and incubated overnight at 4°C with a dilution of the primary antibody against the high concentration of anti-β-actin, anti-p50 antibody and anti-Beclin/Bax/Bcl-2 antibody. β-actin and Lamin B were the internal reference antibodies provided by Sigma [18]. Afterward, the membranes were then incubated with the secondary antibodies (EPITOMICS, Abcam, China) for 2 hours at 4°C, and the signal was read by multi-functional chemiluminescence imaging analyzer (Tanon, 4200SF) and image software with Student’s t test.

### Enzyme-linked immunosorbent assay (ELISA)

Astrocytes cells after 48 h transfection and 24 h reculture were used for the ELISA experiment. The supernatant was collected and assessed for secreted cytokines, including TNF-α, IL-1β, and GAP-43 using the ELISA kit according to the manufacturer’s instructions. In brief, 150 μL of samples were incubated in a 96-well plate coated with primary antibodies for 2 h at RT. After incubation, the samples were washed and incubated with the detection antibody and biotin/streptavidin. Lastly, the plate was read at 450 nm by the microplate reader immediately, then added the STOP solution [19].

### Immunofluorescence

The prepared single-cell suspension was inoculated into a petri-dish with a pre-treated cover glass and then immersed in 100% methanol for 15 minutes. The fixed astrocytes were washed three times in PBS and blocked with 5% serum for 30 minutes. The blocked slice was incubated with a primary antibody (EPITOMICS, Abcam, China) at 4°C overnight and incubated with the secondary antibody (EPITOMICS, Abcam, China) at room temperature for 1 hour. The incubated slice was rinsed with PBST 3 times and each time for 5 minutes [24]. After dropping a drop of sealant on the slice and sealing the tablet, the samples were observed using an inverted fluorescence microscope (Nikon, Tokyo, Japan). Images were captured with Keyence BZ-0023.

### Chromatin immunoprecipitation (CHIP)

Chromatin immunoprecipitation is the only method to study the interaction between DNA and proteins *in vivo*. First, the astrocyte was cross-linked with 37% formaldehyde and broken with ultrasound (VCX750, America). After ultrasonic crushing, the insoluble substance was removed by centrifugation at 10,000× g 4°C for 10 minutes. With 1 μL of antibody as experimental group and without antibody as a control group in the 100 μL sample, the incubated samples were rotated overnight at 4°C. Then 4 μL of 5 M NaCl was added and treated at 65°C for 2 hours to resolve the crosslinking. Next, 60 μl of protein A agarose/NF-κB DNA fragment was added to each tube and was rotated at 4°C for 2 hours. After standing at 4°C for 10 minutes, the samples were centrifuged at 700 rpm for one minute to remove the supernatant. Each tube was eluted with 250 μL of buffer and rotated for 15 minutes at room temperature. After centrifugation, the supernatant was collected and washed repeatedly. The sample tubes were mixed and cross-linked overnight at 65°C after 20 μL of 5 M NaCl was added to each tube [28]. DNA samples were recovered with an omega gel recovery kit, and RT-qPCR analysis was conducted to detect the expression of TWEAK.

RETRACTED

### Statistical analysis

All the determinations were performed at least three times independently. The statistical data were expressed as the mean ± standard deviation (mean ± SD) and analyzed by SAPSS 18.0. Statistical significance was determined with the two-tailed unpaired Student’s t-test and by one-way or two-way analysis of variance (ANOVA) among groups. A value of p < 0.05 was used as criteria for statistical significance.

## Results

We assumed that TWEAK/NF-κB pathway promoted spinal cord injury by inducing astrocyte activation. The effect of the TWEAK-NF-κB axis on SCI and the role of the pro-inflammatory TWEAK/NF-κB pathway in astrocytes after SCI was investigated. TWEAK/NF-κB was a positive correlation feedback loop. TWEAK or NF-κB knockdown inhibited SCI progression in vivo, suppressed the inflammation response of astrocytes after SCI and promoted growth of neurons coincubated with astrocytes after SCI.

### Effects of TWEAK and NF-κB on SCI pathological changes and astrocytes

In this SCI model, the pathological changes of spinal cord injury were analyzed by HE staining and Masson staining. Obvious lesions with bigger cavity areas were found in the model group compared with the control group. Furthermore, the administration of Lv-sh-TWEAK and Lv-sh-NF-κB significantly alleviated the lesion after SCI compared with the Lv-sh-NC groups (Figure S1). The results indicated that TWEAK and NF-κB promoted the SCI progression in vivo. The expression levels of TWEAK/NF-κB on the surface of astrocytes were also detected. RT-qPCR detected higher mRNA levels of TWEAK with sh-nonspecific control. The mRNA levels of TWEAK were reduced effectively after the interference of TWEAK. Similarly, NF-κB should be expressed in various inflammatory tissue and regulate the expression of inflammatory factors and immune-related genes. However, mRNA levels of NF-κB were reduced after the interference of NF-κB (Figure 1(a)). Furthermore, TWEAK induced receptor to reduce astrocyte activity, so astrocyte activity was enhanced after the interference of TWEAK by CCK-8 assay.

RETRACTED

**Figure 1.** Effects of TWEAK and NF-κB on astrocytes. (a) Relative expressions of mRNA-TWEAK and mRNA-NF-κB were confirmed by qRT-PCR assays after the interference of TWEAK or NF-κB in astrocytes. (b) CCK-8 assay analysis of astrocyte viability after the interference of TWEAK or NF-κB. (c) Relative expressions of TNF-α and IL-1β were determined by ELISA after the interference of TWEAK or NF-κB. All the data were represented as mean ± SD, *p < 0.05 and **p < 0.05.

Similarly, when NF-κB was knocked down, the activity of astrocytes was also enhanced, which indicated that NF-κB regulated inflammatory factors and inhibited the proliferation of astrocytes (Figure 1(b)). In addition, astrocytes secrete higher inhibition factors such as TNF-α and IL-1β in this SCI mode. ELISA results showed that levels of TNF-α and IL-1βwere reduced significantly after TWEAK and NF-κB were knocked down (Figure 1(c)). As described above, the primary function of TNF-α was to facilitate the formation of the glial scar, and the primary function of IL-1β was to stimulate astrocytes into an active state by static. Our results revealed that high levels of TWEAK and NF-κB promoted secreting high levels of TNF-α/IL-1β, which affected the inflammation of spinal cord injury.

### Interaction mechanisms of TWEAK and NF-κB

RT-qPCR results showed that the mRNA expression level of NF-κB in the astrocytes reduced in the spinal cord injury mice model after the interference of TWEAK. Similarly, when the NF-κB was knocked down, the mRNA expression level of TWEAK reduced (Figure 2(a)). To further explore the regulating relationship of TWEAK and NF-κB, a western blot (WB) assay was performed by localizing the nucleus with an NF-κB p50 antibody. Results showed that the level of p50 was reduced after the interference of TWEAK (Figure 2(b)). In addition, the CHIP experiment verified that the NF-κB gene regulated the TWEAK gene positively and promoted the expression of TWEAK (Figure 2(c)). CHIP results were consistent with RT-qPCR and WB, which showed that the TWEAK/NF-κB was the positive correlation feedback loop mechanism regulating the proliferation of astrocytes and promoting spinal cord injury.

**Figure 2.** Interaction mechanisms of TWEAK and NF-κB. (a) Relative expression of mRNA-NF-κB and mRNA-TWEAK were confirmed by qRT-PCR assays after the interference of TWEAK or NF-κB in astrocytes. (b) Levels of p50 were detected by western blot analysis. Lamin B was used as the internal reference. (c) Expression of mRNA-TWEAK was confirmed by PCR assay in CHIP. pc: pcDNA3.1 empty vector. pc-NF-κB: pcDNA3.1/NF-κB. All the data were represented as mean ± SD, **p < 0.05 and ***p < 0.001.

RETRACTED

### Effects of TWEAK and NF-κB on autophagy

Autophagy was a double-edged sword in the inflammatory response. On the one hand, autophagy was involved in antigen presentation and promoted inflammatory immune generation; on the other hand, autophagy inhibited inflammatory response by removing the damaged proteins and organelles. This study proved that autophagy-mediated the differentiation and activation of astrocytes, which enhanced the inflammatory response mediating SCI. We observed the process of autophagy and took photographs by electron microscopy as shown in Figure 3(a). The WB results showed that levels of LC3 and Beclin-1 decreased after the interference of TWEAK and NF-κB, in which LC3 and Beclin-1 were the autophagy marker (Figure 3(b)). Immunofluorescence assay showed the same trend as WB assay (Figure 3(c)), which revealed that autophagy was reduced by knocking down TWEAK and NF-κB.

**Figure 3.** Effects of TWEAK and NF-κB on autophagy. (a) Electron micrograph of autophagic cells. (b) Levels of LC3 and Beclin-1 were detected by western blot analysis after the interference of TWEAK or NF-κB. β-actin was used as the internal reference. (c) IF images of LC3 in astrocyte after the interference of TWEAK and NF-κB. All the data were represented as mean ± SD, **p < 0.05.

### Autophagic cell death participated in the effect of TWEAK and NF-κB on astrocytes

Apoptosis and autophagy were two important biological behaviors of cells to maintain homeostasis, which existed not only in the physiological process of normal cells but also in the vital defense mechanism of cells under injury. Apoptosis and autophagy interacted in signal regulation and had many common regulatory elements. Among these regulatory elements, Bax, Bcl-2 and Beclin-1 were independent and closely related, playing a critical regulatory role in apoptosis and autophagy. Lysosome was the essential organelle of autophagy. The number of lysosomes was significantly increased when autophagy activity was enhanced. However, as shown in Figure 4(a), the lysosome number was significantly decreased after TWEAK or NF-κB knockdown compared with the sh-NC groups, while the application of autophagy inducer rapamycin (Rap) reversed the reduction in lysosome number caused by TWEAK or NF-κB knockdown. Increased expression of Bax and Beclin-1 was one typical characteristic of autophagy. After TWEAK and NF-κB were knocked down in astrocytes, WB results showed that Bax and Beclin-1 did not effectively exercise their cross-regulatory effects on apoptosis and autophagy compared the sh-NC groups, while Bcl-2 was significantly up-regulated after silencing TWEAK or NF-κB. After adding Rap, the expression of Bax and Beclin-1 showed an increase compared with the sh-TWEAK or sh-NF-κB groups (Figure 4(b)). CCK-8 assay showed that astrocyte activity was reduced by adding Rap after TWEAK or NF-κB was knocked down (Figure 4(c)). ELISA results revealed that levels of IL-1β and TNF-α were increased by adding Rap after NF-κB or TWEAK was knocked down, promoting inflammation response and spinal cord injury (Figure 4(d)).

RETRACTED

**Figure 4.** Autophagic cell death participated in the effect of TWEAK/NF-κB on astrocytes. (a) Electron micrograph of the lysosome. (b) Expression levels of Bax, Bcl-2 and Beclin-1 were determined by western blot after the interference of TWEAK or NF-κB. β-actin was used as the internal reference. (c) CCK-8 assay analysis of astrocyte viability after the interference of TWEAK or NF-κB and adding Rap. (d) Relative expressions of IL-1β and TNF-α in astrocytes were determined by ELISA after the interference of NF-κB or TWEAK and adding Rap. All the data were represented as mean ± SD, **p < 0.05, ***p < 0.001, ^#^p < 0.05 and ^##^p < 0.01.

### Effect of TWEAK and NF-κB on co-cultured neurons

Neuronal apoptosis was a critical factor in secondary injury after spinal cord injury. Apoptotic cells were found in any injured spinal cord and detected at sites and even at peripheral segments in almost all types of cells. Cells of the nervous system were mainly composed of neurons and glial cells. Glial cells provide nutrients to neurons, and their synapses connect capillaries with neurons directly. However, if large numbers of glial cells died or overgrew, the growth of neurons would be adversely affected. Through the ELISA experiment, we found that levels of TNF-α and IL-1 βsecreted by neurons were reduced after the interference TWEAK and NF-κB (Figure 5(a)). We thus further characterized the expression of growth-associated protein-43 (GAP-43), a kind of neuro-specific protein involved in the growth of nerve cell synapses and regeneration. The results of WB assays showed that the expression of GAP-43 was significantly enhanced after the interference of TWEAK and NF-κB (Figure 5(b)), which suggested that restraining the excess growth of astrocytes was beneficial to the growth of neurons. Likewise, interference of TWEAK and NF-κB enhanced the expression of GAP-43 secreted by neurons as determined by immunofluorescence analysis, and the trend was consistent with WB (Figure 5(c)).

RETRACTED

**Figure 5.** Effect of TWEAK/NF-κB on co-cultured neurons. (a) The relative expression values of TNF-α and IL-1β in the co-cultured neurons were determined by ELISA after the interference of TWEAK or NF-κB. (b) The expression level of GAP-43 was determined by western blot after the interference of TWEAK or NF-κB. β-actin was used as the internal reference. (c) IF images of GAP-43 in the co-cultured neurons after the interference of TWEAK or NF-κB. All the data were expressed as the means ± SD. *p < 0.05 and **p < 0.05.

### Autophagic cell death was involved in the effect of TWEAK and NF-κB on co-cultured neuron

To further understand the implications of autophagic cell death in the effect of TWEAK/NF-κB on the co-cultured system, we analyzed the expression of TNF-α, IL-1β and GAP-43 in these astrocytes co-cultured neurons. ELISA results showed that levels of TNF-α and IL-1β in neurons increased obviously after adding Rap, promoting inflammation and SCI (Figure 6(a)). Besides, increased generation of GAP-43 was observed after the interference of TWEAK and NF-κB as determined by WB analysis (Figure 6(b)). However, large numbers of astrocytes died after adding Rap into the co-culture system because of an adverse effect on the growth of neurons (Figure 6(b)). Consistent with our findings as mentioned above, immunofluorescence assay of Gap-43 in neurons conformed to WB results (Figure 6(c)).

**Figure 6.** Autophagic cell death was involved in the effect of TWEAK/NF-κB on astrocytes co-cultured neurons. (a) Relative expressions of TNF-α and IL-1β in the co-cultured neurons were determined by ELISA after the interference of TWEAK/NF-κB and adding Rap. (b) Expression levels of GAP-43 in the co-cultured neurons were determined by western blot after the interference of TWEAK or NF-κB and adding Rap. β-actin was used as the internal reference. (c) IF images of GAP-43 in the co-cultured neurons after the interference of TWEAK or NF-κB and adding Rap. All the data were expressed as the means ± SD. ***p < 0.001 and ^##^p < 0.01.

## Discussion

At present, the detailed signaling pathway of astrocyte promoting SCI is still unclear. Therefore, it is important to explore the function and mechanism of upstream regulatory gene pathway on the secretion of related proteins in astrocytes and the progression of SCI. These studies might be conducive to the targeted selection of treatment strategies to reduce injury and restore neurological function. Various factors secreted by astrocytes play different roles in different microenvironments or concentrations after spinal cord injury, which may be either simulative or inhibitory [17,29]. However, the mechanisms of feedback loop regulating astrocytes to aggravate SCI remain to be explored. For example, how to change the static state of astrocytes into an activated state or even into the proliferative state after SCI; How factors secreted by astrocytes affect the microenvironment of the damaged area; How to regulate a series of cytokines secreted by astrocytes after SCI, including neuroactive factors and neuroinhibitory factors.

RETRACTED

TWEAK is a multifunctional cytokine that can promote inflammation, angiogenesis and regulate cell growth, development and apoptosis. Studies have shown that TWEAK is involved in a variety of inflammatory and autoimmune diseases, such as atherosclerosis, heart failure, the pathogenesis of chronic kidney disease, II type diabetes. In particular, TWEAK is found to promote persistent NF-κB activation in mouse tubular epithelial cells. In tubular epithelial cells, TWEAK induces B phosphorylation and RelA nuclear translocation through Fn14, thus enhancing NF-κB binding to DNA and transcriptional activity. In this work, we brought new insights on the regulatory mechanism of the TWEAK/NF-κB axis in mouse astrocytes after SCI and demonstrated that this new feedback loop might be involved in astrocyte proliferation and SCI inflammatory disease [30,31].

Meanwhile, increasing attention has been attracted to the tumor necrosis factor receptor (TNFR) family. TNFR family participated in cell apoptosis and other types of programmed cell death widely caused by an inflammatory reaction and lymphocyte activation. These receptors produced different signaling responses according to the different cell types and environmental factors. Diana Spicarova e*t al*. have reported that the expression of TNFR is not clearly detected in the normal spinal cord. In contrast, the expression levels of TNFR1 were detected in normal DRGn afferent fibers of the spinal cord and thin layer area I and II after spinal cord, but there is no evidence for the existence of TNFR2 [32].

Inflammatory cytokines have been confirmed to mediate reactive astrocyte proliferation in neurodegenerative diseases, such as TNF-α and IL-1β. In the context of those findings, our experiment established a SCI model for this TWEAK/NF-κB signaling pathway which resulted in changes of the TNF-α/IL-1β expression level in astrocytes after SCI. Here, we investigated how the TWEAK/NF-κB axis signaling influenced the normal function of astrocytes or neurons and the correlation between two genes, thus revealing this regulatory mechanism promoting SCI. We firstly identified the effects of TWEAK and NF-κB on astrocytes through the interference of TWEAK and NF-κB, and the results revealed that lower levels of TWEAK/NF-κB reduced secreting TNF-α/IL-1β. Similarly, Kim *et al*. found that NF-kB activation by the TLR5-Nox4 axis leads to the expression of proinflammatory cytokines, including TNF-α, IL-1β and IL-6 [33]. By activation of its receptor Fn14, TWEAK stimulates the production of proinflammatory cytokines (TNF-α, IL-1β and IL-6) and chemokines in a variety of cell types [34,35].

RETRACTED

We further investigated the effects of autophagic cell death on astrocytes through TWEAK/NF-κB signal pathway, resulting in the impact of promoting inflammation and SCI after TWEAK/NF-κB were knocked down. In addition, we demonstrated the effect of TWEAK/NF-κB knocked down in the co-culture system of astrocytes and neurons. Together, our findings suggested the importance of TWEAK/NF-κB in astrocytes, which had the effect of promoting inflammation of SCI.

## Conclusions

The findings of this study indicated that TWEAK and NF-κB might act as a positive modulator of SCI by inducing astrocyte activation signaling axis, suggesting that the TWEAK/NF-κB feedback loop exerted multiple effects on SCI through the astrocyte activation response. In this work, we brought new insights on the regulatory mechanism of TWEAK/NF-κB axis in mouse astrocytes and provided evidence that this new feedback loop might be involved in astrocyte proliferation and SCI inflammatory disease.

## Supplementary Material

Supplemental Material

## Data Availability

All data generated or analysed during this study are included in this published article.
